The article "TGF-β1 Induces Interlukin-11 Expression and Pro-Fibrotic Effect by DNA Demethylation in Subconjunctival Fibroblasts" was retracted in 2023. Reasons: signs of a paper mill; suspected computer-generated content; unreliable results or conclusions; concerns about the data.

# TGF-*β*1 Induces Interlukin-11 Expression and Pro-Fibrotic Effect by DNA Demethylation in Subconjunctival Fibroblasts

**DOI:** 10.1155/2022/7729827

**Published:** 2022-07-12

**Authors:** Shuhao Fu, Zhaozeng Lu, Wen Ye

**Affiliations:** Department of Ophthalmology, Huashan Hospital, Fudan University, Shanghai 200040, China

## Abstract

**Objective:**

To assess Interlukin-11 (IL11) expression in the tears of patients after filtration surgery and to find out its pro-transdifferentiational and pro-fibrotic functions and mechanisms on subconjunctival human Tenon's capsule fibroblasts (HTFs) induced by transforming growth factor beta1 (TGF-*β*1).

**Methods:**

Tears were collected from glaucoma patients with or without filtration surgery. The expression of IL11 in tears was examined by enzyme-linked immunosorbent assay. Primary HTFs were prepared as an expansion culture of human Tenon's explants from patients undergoing cataract surgery. TGF-*β*1 and IL11 were used to stimulate the cultured HTFs. Quantitative RT-PCR and western blot analyzed the roles of TGF-*β*1 in IL11 and DNA methyltransferase (DNMT) expression and the effects of IL11 on collagen-1A1 and *α*-smooth muscle actin expression. The effects of IL11 on human HTFs' migration were tested via the scratch-wound assay. MassARRAY platform of Sequenom was applied for analyzing the quantitative methylation of the IL11 promoter region.

**Result:**

Our data presented significantly high levels of IL11 in the tears of patients who underwent filtration surgery with uncontrolled intraocular pressure (IOP) compared with those who underwent filtration surgery with controlled IOP. The up-regulation of IL11 was related to TGF-*β*1. We also found that TGF-*β* induced IL11 up-regulation in the HTFs, which activates the HTFs and enhanced the translation of the pro-fibrotic protein expression. This is correlated with inhibiting the activity and expression of DNMTs and demethylating the IL11 promoter. Therefore, IL11 may be an ideal target to be regulated to control the filtering pathway scar formation.

## 1. Introduction

Glaucoma is the commonest reason of irreversible blindness worldwide [1]. The major choice for patients to treat uncontrollable intraocular pressure (IOP) is filtration surgery [2]. However, the scarring of the filtering pathway after operation seriously affects the success rate and patients' quality of life [3]. No safe and effective drugs can be used to control the filtering pathway scar formation so far. The main cellular component in the filtering scar tissue is human Tenon's capsule fibroblast (HTFs). It has come to light that transforming growth factor beta1 (TGF-*β*1)-induced transdifferentiation of the HTFs to alpha smooth muscle activin (*α*-SMA)-positive myofibroblasts (MFs) is one of the most vital events worldwide for postoperative scar formation and healing [4]. Since TGF-*β*1 has multiple effects in both physiological and pathological conditions, blocking TGF-*β*1 or its receptors may have other side effects. Therefore, the exploration of its downstream mechanism helps find safer and more specific inhibitory targets, which is of great significance in finding new therapeutic strategies and drug targets.

Interleukin 11 (IL11) has been confirmed to be the downstream of the TGF-*β*1 signaling pathway in several fibrosis-related studies. IL11 plays a key role in mediating fibroblasts' transdifferentiation and tissue fibrosis [5]. DNA methylation, catalyzed by DNA methyltransferases (DNMTs), is one of the epigenetic regulatory mechanisms significantly affecting gene expression. A study has proven that HTFs' transdifferentiation and fibrosis can be induced by DNA hypomethylation [6]. It is found in human primary fibroblasts in oral wound healing that inhibiting DNA methylation allows TGF-*β*1-induced IL11 expression, which shows the mechanism of how TGF-*β*1 regulates IL11 [7]. In this study, IL11 was obviously elevated in the tears of patients with failed filtration surgery. Our results also showed that TGF-*β*1 induced IL11 up-regulation in the HTFs, which activates the HTFs and enhanced the translation of the pro-fibrotic protein expression. This was caused by suppressing the expression and activity of DNMTs and demethylating the IL11 promoter. Therefore, IL11 plays an important role in TGF-*β*1-mediated filtering pathway fibrosis. IL11 may be an ideal target to be regulated to control the filtering pathway scar formation.

## 2. Materials and Methods

Huashan Hospital Institutional Review Board approved both tear and human Tenon's capsule tissue collection for cell culture trials, and all procedures met the requirements of the Declaration of Helsinki. Besides, this article was performed after obtaining the consent of all subjects.

### 2.1. Tear Collection and Analysis

Tear samples were obtained non-traumatically from the inferior tear meniscus. 5 *μ*L of tear was collected with glass capillary micropipettes. Tear samples were immediately eluted fully and then collected into a sterile collection tube. During collection, the tube was kept cold (4°C), and after collection, it was placed at the temperature of −80°C until the activity assays were performed. The concentrations of IL11 in the tears were analyzed using a Human IL-11 ELISA Kit (ELH-IL11, RayBiotech, USA).

### 2.2. Cell Culture

Patients receiving cataract surgery provided human Tenon's explants. Among the subjects, there were two females and one male (age: 58–65 years) without glaucoma or ocular surgery history. Primary HTFs were cultured for an expansion of the human Tenon's explants. Specifically, a Dulbecco's modified Eagle's medium (DMEM, Hyclone, Logan, UT, USA) with 100 U/mL penicillin, 10% heat-inactivated fetal bovine serum (FBS, Gibco, Life Technologies, Grand Island, NY, USA), and 100 g/mL streptomycin (Biochrom, Berlin, Germany) was prepared for culturing primary HTFs. The cells in the logarithmic growth phase were maintained. This paper adopted cells from passages 5 to 10 for all trials. The culture in monolayers was performed at 37°C for the fibroblasts from the same initial colony, and the medium was displaced every 3 days.

### 2.3. TGF-*β*1, 5-Aza-dc, SB-431542, and IL11 Treatments

A six-well plate was utilized to culture HTFs with a concentration of 5 × 10^4^ HTFs/mL. After the completion of preparation at 10 *µ*g/mL in PBS with 0.1% bovine serum albumin (BSA), human recombinant stock solution TGF-*β*1 (PeproTech, Rocky Hill, NJ, USA) was conserved at −20°C. Later, the solution was diluted into 10 ng/mL using DMEM for subsequent cultures. Additionally, 50 *µ*g/*μ*L of 5-Aza-dc (Sigma-Aldrich, St. Louis, MO, USA) was prepared in ddH_2_O as a stock solution and stored at −80°C under the condition of light avoidance. Then the solution was put to the culture system at different final concentrations of 5 *μ*M. After being diluted in dimethyl sulfoxide (DMSO), 5 mM of SB-431542 was stored at −20°C, and then cultured at a final concentration of 5 *μ*M. The stock solution of IL11 (PeproTech, Rocky Hill, NJ, USA) at 10 *µ*g/mL was prepared using PBS with 0.1% bovine serum albumin (BSA), and then stored at −20°C. Next, the solution was diluted with DMEM and cultured with 5 ng/mL as a final concentration. For research more than 12 h, the culture medium was altered by a fresh one containing the identical compound (s) every 12 h.

### 2.4. Scratch-Wound Assay

Cell migration activity was evaluated by the scratch-wound assay, and it is a section of the scarring process. Firstly, we used 6-well plates with poly-D lysine (100 *μ*g/L) coated for the growth of the HTFs (5 × 10^4^/well). Serum-free DMEM replaced the culture medium for 24 h to synchronize cell growth. After sterilization, a 1 mL pipette tip was used to scrape the confluent monolayer of the HTFs to avoid cell gaps. Upon washing by PBS, the HTFs were treated with 5 ng/mL IL11 or DMEM or 10 ng/mL TGF-*β*1. The denuded area of the HTFs with IL11 or TGF-*β*1 treatment were imaged by phase contrast microscope and quantified by ImageJ software (1.48 v, Wayne Rasband, National Institutes of Health, USA) at 24 h after scratch and normalized to the denuded area at 0 h. A masked researcher was responsible for the image analysis.

### 2.5. Nuclear Extraction and DNA Methyltransferase Activity Assay

After 24 h serum starvation, the HTFs were treated with 10 ng/mL of TGF-*β*1 for 0, 24, and 48 h. The nuclear extraction kit from Sangon (Shanghai, China) was used to prepare nuclear extracts following related instructions. BCA Protein Assay Reagent Kit (Pierce, Rockford, IL, USA) was utilized to check the protein concentration in line with the manual. About 20 *μ*g of nuclear protein of each sample was collected for activity assay. EpiQuik DNA Methyltransferase Activity Assay Kit from Epigentek (Farmingdale, NY, USA) was employed for DNA methyltransferase activity assessment and the outcomes were calculated in light of the user guide.

### 2.6. Quantitative Real-Time PCR

TRIzol reagent (Ambion, Life Technologies, Carlsbad CA, USA) was adopted for the total RNA extraction of each sample on the basis of the instructions, and spectrophotometry for quantification. Using 1 *µ*g total RNA extract, first-strand cDNA with a final volume of 20 *µ*L was synthesized (M-MLV Reverse Transcriptase; ImproII; Promega, Mannheim, Germany) at 42°C. RNA translation and extraction of the HTFs to the cDNA were conducted as introduced herein. Subsequently, quantitative real-time RT-PCR (RT-qPCR) was implemented using 2 × SYBR Premix Ex Taq™ II (Takara, Japan) with the ABI 7500 System (Applied Bio-systems, Foster City, CA, USA). The software Primer 5.0 (Premier Software, Palo Alto, CA, USA) was used for specific primer design, and Biotnt (Shanghai, China) for sequence manufacture as displayed in Table 1 [6]. The target gene expression level of each sample was normalized to the GAPDH transcript level.

### 2.7. Western Blot Analysis

PBS buffer was used twice for washing cells in 6-cm dishes; 100 *µ*L of RIPA buffer (Beyotime Biotech, Shanghai, China) with a protease inhibitor cocktail (Roche, Mannheim, Germany) for cell lysis; BCA Protein Assay Reagent Kit (Pierce) for protein concentration measurement of each sample; and a 10% SDS-PAGE gel for protein (20 *μ*g/lane) resolving were utilized as well. After electrophoresis separation, a nitrocellulose membrane (Millipore, Billerica, MA, USA) was prepared for protein extract transferring. Later, the membrane was blocked and evaluated with primary antibodies against DNMT1 (1 : 500, Cell Signaling Technology, Danvers, MA, USA), DNMT3a (1 : 500, Cell Signaling Technology), *α*-SMA (1 : 1000, Sigma), DNMT3b (1 : 500, Abgent, San Diego, CA, USA), GAPDH (1 : 1000, Cell Signaling Technology), and Col1A1 (1 : 100, Santa Cruz). Goat anti-rabbit or goat anti-mouse IRDye secondary antibodies were utilized for revealing bound antibodies; Li-COR Odyssey system (LI-COR, Lincoln, NE, USA) was used for visualization; and Image J software (National Institutes of Health, USA) was utilized for signal analysis. Based on the GAPDH band, the normalization of the band density of each protein was performed.

### 2.8. DNA Methylation Analysis

Wizard SV Genomic DNA Purification System (Promega, WI, USA) was in charge of genomic DNA extraction from the cultured cells in line with the manufacturer's illustration. According to the absorbance at 260 and 280 nm, the DNA's purity and concentration were determined. Following the instructions, 1 *µ*g of bisulfite-treated genomic DNA from each sample was implemented through the EZ DNA methylation kit (Zymo Research, CA, USA). Sequenom MassARRAY platform (CapitalBio, Beijing, China), combined with RNA base-specific cleavage and composed of matrix-assisted laser desorption/ionization time-of-flight (MALDI-TOF) mass spectrometry, was utilized for the quantitative analysis of IL11 methylation (Gen-Bank Accession Number: NM_000641). Methprimer (https://www.urogene.org/methprimer/) was included for PCR primer design. For designing the primer systems used in the methylation analysis, T7-promoter-tagged reverse primer was used to acquire suitable products for transcription in vitro, and 10mer-tagged forward primer for the PCR balance. The primers on the basis of the reverse complementary strands of the IL11-promoter applied in this paper are shown as follows (5′-aggaagagagTTTTTTTTAATTTTTTTAATTTTTTTT-3′ and 3′-cagtaatacgactcactatagggagaaggct TAAATCCCTCTCCTCCCTACCT-5′). MassARRAY Compact MALDI-TOF MS (Sequenom) was adopted to obtain the mass spectra and the Epityper software version 1.0 was used to generate the methylation ratios (Sequenom).

### 2.9. Statistical Analysis

All outcomes were expressed as mean ± standard deviation (SD). With SPSS 19.0 software (SPSS, Inc., Chicago, IL, USA), one-way ANOVA was performed for statistical analyses; unpaired *t*-test was used for comparisons between two groups; and Fisher's least significant difference test was performed for comparisons among three or more groups. *P* < 0.05 is significantly different.

## 3. Results

### 3.1. Patients and Clinical Outcomes

Sixteen eyes from 16 patients were involved in this research (Table 2). Four healthy subjects served as the control group with a mean age of (50.5 ± 6.7) years. The other 12 subjects were patients who received different operations. Four glaucoma patients underwent filtration surgery with controlled IOP and served as the F1 group, four glaucoma patients underwent filtration surgery with uncontrolled IOP and served as the F2 group, and four patients underwent cataract extraction and served as the C group. Their mean age was (56.5 ± 8.9) years; (50.75 ± 6.4) years; and (63.0 ± 8.8) years, representative with no statistically significant differences. Their IOP was measured and is shown in Figure 1(a). The concentrations of IL11 in tears from different groups are shown in Figure 1(b). We found elevated IOP in the F2 group which indicated filtration scar formation. Significant elevation of tear IL11 level was also found in those patients with failed filtration surgery compared to not only patients in the control group but other operated patients as well.

### 3.2. TGF-*β*1 and DNMT Inhibitor Up-Regulate the mRNA and Protein Expressions of IL-11 in the HTFs

Using 10 ng/mL TGF-*β*1 can induce the transdifferentiation of the HTFs and cause the fibrosis effect as described before [8], which can be used as a cell model of the filtration pathway scar formation. IL11 is also proved to be the downstream of TGF-*β*1-induced fibroblasts' transdifferentiation and tissue fibrosis in other tissues. Thus, we tested if TGF-*β*1 could induce IL11 expression in the HTFs. We found that treating with TGF-*β*1 significantly up-regulated IL11 at the mRNA level via RT-qPCR since 12 h (Figure 2(a)). After measuring IL11 protein in the supernatant of the HTFs with the ELISA assay, gene expression changes were checked at the protein level (Figure 2(b)). We also found that the DNMT inhibitor, 5-Aza-dc, induced DNA hypomethylation, which may relate to the HTFs' transdifferentiation [6]. Herein, the HTFs were treated with 5-Aza-dc (5 *μ*M), and TGF-*β*1 with or without 5-Aza-dc. Treating with 5-Aza-dc could also up-regulated IL11 levels in the HTFs on both protein and mRNA levels (Figures 2(c) and 2(d)). The IL11 elevation was strengthened when treated with 5-Aza-dc and TGF-*β*1.

### 3.3. IL11 Activates HTFs and Drives Fibrosis

Since research showed that IL11 plays a key role in mediating fibroblasts' transdifferentiation and tissue fibrosis, we evaluated if changes in the HTFs indicative of fibrosis could be induced by IL11. HTF migration is regarded as one of the momentous biological events in subconjunctival wound healing. Therefore, the scratch-wound assay was enrolled to determine the function of IL11 in the HTFs' migration. We created a denuded area by tip scratching in the confluent monolayer of the HTFs. The denuded area in the HTFs treated with 5 ng/mL IL11 or 10 ng/mL TGF-*β*1 was imaged and quantified at 24 h after scratch (Figure 3(a)). A notable decrease was observed in IL11-treated HTFs in the denuded area at 24 h in comparison with that at 0 h in the same area of the TGF-*β*1-treated group (Figure 3(b)). Then, we treated the HTFs with 5 ng/mL IL11 for 24 h. Exposure to IL11 revealed a significant increase in *α*-SMA protein levels but not in the mRNA level which was different from TGF-*β*1. Meanwhile, IL11 also up-regulated the extracellular matrix, Col1A1, expression only at the protein level (Figures 3(c)–3(f)). It is surprising that IL11 activates the HTFs and drives fibrosis mainly at the post-transcription level.

### 3.4. TGF-*β*1 Inhibits the DNMT Activity and Expression

Since TGF-*β*1 and 5-Aza-dc can both up-regulate IL11 in the HTFs, we tested if TGF-*β*1 could inhibit the DNMT expression and activity in the HTFs. Global DNMT activity level was tested using fresh nuclear extracts, and we found that TGF-*β*1 gradually inhibited the DNMTs' activity in the HTFs since 6 h (Figure 4(a)). Besides, compared with the control group, treatment with TGF-*β*1 obviously declined DNMT3a and DNMT1 expression in the HTFs' group (Figures 4(b)–4(d)). Nevertheless, up to 48 h, DNMT3b expression was not affected by TGF-*β*1 treatment (Figures 4(c) and 4(d)). DNMT1 and DNMT3a expressions' down-regulation was lagged behind the decrease in the activity. These outcomes suggested that the occurrence of the up-regulation of IL11 expression lagged behind the time course of the DNMT activity and expression decrease, indicating that TGF-*β*1-induced up-regulation of IL11 may relate to DNA demethylation in the IL11 promoter.

### 3.5. TGF-*β*1 Induces DNA Demethylation in the IL11 Promoter Region

According to the previous results, we proved that TGF-*β*1 up-regulated IL11 in the HTFs. TGF-*β*1 also gradually suppressed the DNMTs' activity and expression in the HTFs. The onset of the up-regulation of IL11 expression lagged behind the time course of the DNMT activity and expression decrease. Therefore, we tried to figure out if TGF-*β*1 induced the expression of IL11 by promoter demethylation. The HTFs were treated with 10 ng/mL TGF-*β*1 for 24 h. Genomic DNA extraction was conducted and the extracts were subjected to bisulfite sequencing analysis. In addition, we analyzed the DNA fragment from the IL11 promoter including one CpG island, evaluated the methylation level of each CpG site within this region, and divided the 14 CpG sites in the promoter region into 9 CpG site units.  Figure 5 shows that, after 24 h incubation, TGF-*β*1 obviously reduced the methylation percentage across multiple CpG sites. Demethylation changed a lot (22% of the level from the control samples) from the 6^th^ to the 14^th^ CpG sites, while for the other CpG sites, no obvious change could be observed.

## 4. Discussion

IL11 belongs to the family of interleukin-6 (IL6) cytokines [9]. The relation between IL11 and fibrosis was first reported in 1996 and stated that recombinant human IL11 induces bone marrow fibrosis (myelofibrosis) [10]. Afterwards, IL11 gain of function was fully discovered. It was found in the lungs of patients with idiopathic pulmonary fibrosis that IL11 expression level correlates with the severity of lung fibrosis [11]. IL11 is also found elevated in the serum of patients with systemic sclerosis [12]. Herein, we found that glaucoma patients who underwent filtration surgery with uncontrolled IOP had elevated IL11 expression in their tears compared to patients undergoing filtration surgery with controlled IOP. This finding indicates that IL11 may also exert a vital function in the filtering pathway scar formation.

It is proved that TGF-*β* is released in the subconjunctival tissue after filtration surgery which results in HTFs' transdifferentiation and the start of wound healing [13, 14]. The continuous release of TGF-*β* leads to further fibroblasts' migration, proliferation, and synthesis of extracellular matrix which causes scar formation and surgical failure [15, 16]. The key role of IL11 in TGF-*β*1-mediated fibroblast transdifferentiation and tissue fibrosis has been proven in many fibrosis-related studies [5, 17, 18], and may even be the central regulator factor of fibrosis [19, 20]. In cardiovascular fibrosis and kidney fibrosis studies, TGF-*β*1-induced primary human fibroblasts showed elevated IL11 expression. IL11 up-regulation was also found in hepatic stellate cells after incubation with TGF-*β*1 using RNA-Seq analysis which was confirmed at the protein level [18]. Our outcomes exhibited that TGF-*β*1 significantly up-regulated IL11 at both the mRNA level via RT-qPCR and the protein level using an ELISA assay which is in keeping with previous data on fibroblasts from other organs.

Using recombinant human IL11, cardiac fibroblasts were activated, which led to extracellular matrix production and invasion. In mice, fibroblast-specific IL11 over-expression or recombinant mouse IL11 injection can lead to heart and renal fibrosis which causes organ failure [5, 17]. These results all showed the pro-fibrotic effect of IL11. Our experiments also demonstrated that IL11 activates the HTFs and drives fibrosis. The scratch-wound assay showed an enhanced migration rate in the HTFs treated with IL11. Meanwhile, the markers of transdifferentiation and extracellular matrix synthesis were also significantly elevated in IL11-treated HTFs. However, surprisingly, the pro-fibrotic effect of IL11 is only shown at the protein level and not related to transcriptional changes, which corresponds with the findings in cardiac fibroblasts [5].

It is noticed that the up-regulation of IL11 is the dominate transcriptional response to TGF-*β*1 exposure. We wondered how TGF-*β*1 induced IL11 up-regulation in the HTFs. 5-Aza-dc, a cytidine chemical analogue, can inhibit DNMT and lead to genome-wide DNA methylation decrease. Our previous study highlighted that 5-Aza-dc-induced DNA hypomethylation relates to HTFs' transdifferentiation [6]. Herein, we found that 5-Aza-dc had a similar effect on IL11 regulation as TGF-*β*1 did, indicating an additional mechanism that TGF-*β*1 regulated the IL11 gene expression by suppressing DNA methylation.

DNA methylation is a kind of epigenetic regulation which is catalyzed by DNMTs [21]. Instead of changing the nucleotide sequence, DNA methylation directly modifies genomic DNA and affects gene expression. The regulation of the DNMTs' activity and expression can directly affect the genomic DNA methylation level and target gene expression [22, 23]. In our research, TGF-*β*1 was observed to markedly suppress the global DNMT activity and down-regulate the mRNA and protein expressions of DNMT1 and DNMT3a in a time-dependent manner. Our outcomes correspond with the findings in the reports on rat lung fibroblasts [24] and cardiac fibroblasts [25]. Additionally, the onset of the up-regulation of IL11 expression lagged behind the time course of the DNMT activity and expression decrease, indicating that TGF-*β*1-induced up-regulation of IL11 may relate to DNA demethylation in the IL11 promoter region.

Genomic hypermethylation is observed most commonly in CpG islands in gene regions, while in cancer, hypomethylation is seen frequently in both moderately and highly repeated DNA sequences [26]. Some scholars have provided evidences that methylation at the CpG sequence in the promoter region suppresses gene expression and vice versa. In this report, DNA fragments from the IL11 promoter region were analyzed. Our results showed that TGF-*β*1 could greatly decrease the methylation percentage across multiple CpG sites in the IL11 promoter and enhance its expression. Similar findings in human gingival fibroblasts showed DNA demethylation supports TGF-*β*-induced IL11 expression [7]. This might be the possible mechanism of how TGF-*β*1 induced IL11 up-regulation and fibrosis effect in the HTFs (Figure 6). Further study is needed to focus on the downstream signaling pathway activated by IL11 in the HTFs.

## 5. Conclusion

Taken together, TGF-*β*1 induced IL11 up-regulation in the HTFs which activates the HTFs and enhanced the translation of pro-fibrotic protein expression. This is correlated with inhibiting the activity and expression of DNMTs and demethylating the IL11 promoter. Therefore, IL11 may be an ideal target to be regulated to control the filtering pathway scar formation.

## Figures and Tables

**Figure 1:** The concentrations of tear IL11 level from patients with or without surgery. (a) IOP measurement in patients who underwent different surgeries. (b) ELISA tests of IL11 level in patients' tears of the corresponding groups. Data are mean and SD, ^*∗∗*^*P* < 0.01 vs. Control, ^##^*P* < 0.01 vs. F1 group, ^++^*P* < 0.01 vs. C group. (F1 group represents patients who underwent filtration surgery with controlled IOP; F2 group represents patients who underwent filtration surgery with uncontrolled IOP; C group represents patients who underwent cataract extraction).

**Figure 2:** TGF-*β*1 and DNMT inhibitor can up-regulate the mRNA and protein expressions of IL11 in the HTFs. (a) The HTFs were treated with 12 h serum starvation followed by 10 ng/mL TGF-*β*1 for 0, 12, and 24 h; RT-qPCR was utilized to determine the expression change of IL11. (b) ELISA tests of IL11 protein expression in the supernatant of the HTFs after TGF-*β*1 treatment. (c) The HTFs were serum-starved for 12 h and then treated by 5-Aza-dc (5 *μ*M), TGF-*β*1 (10 ng/mL), and TGF-*β*1 together with 5-Aza-dc for 24 h. A DMEM-alone group was included as a control. RT-qPCR was adopted for assessing the changes in the expressions of IL11. (d) ELISA tests of IL11 protein expression in the supernatant of the HTFs of the corresponding groups. Data were SD and mean from three independent examinations, each with triplicate samples. ^*∗∗*^*P* < 0.01, ^*∗∗∗*^*P* < 0.001 vs. 0 h value. ^##^*P* < 0.01, ^###^*P* < 0.001 vs. control group at the same time point by one-way ANOVA followed by the Fisher test (T represents TGF-*β*1; 5A represents 5-Aza-dc).

**Figure 3:** IL11 activates the HTFs and leads to the pro-fibrotic effect mainly at the protein level. The denuded area was created by tip scratching in the HTFs' confluent center region. The HTFs were treated with 10 ng/mL TGF-*β*1 or 5 ng/mL IL11 for 0, 12, and 24 h, and then photographed. (a) Typical images at different time points for the different treatment groups after scratch. Scar bar = 500 *μ*m. (b) The percentages of the denuded area (denuded area at the specified time point/denuded area at 0 h) were analyzed quantitatively after different treatments at different times. The HTFs were treated with 10 ng/mL TGF-*β*1 or 5 ng/mL IL11 for 24 h after 12 h serum starvation. A DMEM-alone group was included as a control. ^*∗*^*P* < 0.05, *vs*. their respective 0 h value. (c-d) RT-qPCR was employed for checking the changes in the expressions of the transdifferentiation marker *α*-SMA (c) and extracellular matrix Col1A1 (d). (e-f) Western blot analysis of the expression of *α*-SMA and Col1A1 proteins. Data were mean and SD of three independent tests, triplicate samples for each. ^#^*P* < 0.05, ^##^*P* < 0.01*vs*. Control by one-way ANOVA and then by the Fisher test.

**Figure 4:** TGF-*β*1 induces changes in the DNMT activity and expression in the HTFs. (a) Upon serum starvation for 12 h, the HTFs were treated with 10 ng/mL TGF-*β*1 for 0, 6, 12, and 24 h. The global DNMT activity was analyzed by a DNMT activity assay kit. The DNMT activity in the TGF-*β*1-treated HTFs was much lower than that in the control (*n* = 3). (b) Expression changes in the DNMTs over different time periods assessed by RT-qPCR. (c) Typical pictures of western blots of DNMTs at 0, 6, 12, and 24 h after TGF-*β*1 treatment of the HTFs. (d) DNMT1, DNMT3a, and DNMT3b protein levels in the HTFs after TGF-*β*1 treatment. Data were average value and SD from three independent trials, triplicate samples for each. ^*∗*^*P* < 0.05, ^*∗∗*^*P* < 0.01, ^*∗∗∗*^*P* < 0.001 vs. 0 h by one-way ANOVA and the Fisher test.

**Figure 5:** TGF-*β*1 induces DNA demethylation in the IL11 promoter region. After 12 h serum starvation, the HTFs were treated by 10 ng/mL TGF-*β*1 for 24 h. A DMEM-alone group was included as a control. The methylation ratios of the 14 CpG sites in the IL11 promoter region were obtained by MassARRAY Platform. (a) DNA fragments from human IL11 promoter region was amplified for the analysis of the methylation level. The fragments were labeled as the promoter region sequence. The location of the promoter region (−1572 bp to −1304 bp) and one CpG island were represented by a blue bar and a green bar, respectively. In light of the reverse complementary strands of these fragments, PCR primer design was performed. The promoter region sequence indicated 269 bp fragments and the CpG sites were counted from 1 to 14 from the 3′- end to the 5′-end. (b) Quantitative methylation levels are shown in a color scale from red to light yellow which represent the methylation level from 0% to 100%, while the grey circle represents missing data. (c) Average methylation levels of the CpG sites in the IL11 promoter region. Data were SD and mean from four independent tests. ^*∗*^*P* < 0.05, ^*∗∗*^*P* < 0.01*vs*. control group at the same CpG site by one-way ANOVA followed by the Fisher test (C represents Control; T represents TGF-*β*1).

**Figure 6:** Possible mechanism of TGF-*β*1 inducing IL11 promoter demethylation that evokes HTF transdifferentiation and fibrosis.

**Table 1:** Primer sequences.

Target gene	Forward primer (5′-3′)	Reverse primer (5′-3′)
IL-11	GACCTACTGTCCTACCTGCG	AGTCTTCAGCAGCAGCAGTC
*α*-SMA	CCGACCGAATGCAGAAGGA	ACAGAGTATTTGCGCTCCGAA
COL1A1	AGGGCCAAGACGAAGACATC	GTCGGTGGGTGACTCTGAGC
DNMT1	CCTCATCGAGAAGAATATCG	GGATCCATCAGAATGTATTC
DNMT3a	TATTGATGAGCGCACAAGAGAGC	GGGTGTTCCAGGGTAACATTGAG
DNMT3b	GAAGGGGTGTGCTGAGTT	GGGTTTGAGGGGGTGTCTT
GAPDH	GGGAAGGTGAAGGTCGGAG	GGGGTCATTGATGGCAACA

**Table 2:** Basic clinical characteristics of the participants.

Group	Group classification	Number	Age	Disease status
	F1	4	56.5 ± 8.9	Underwent filtration surgery with controlled IOP
	F2	4	50.75 ± 6.4	Underwent filtration surgery with uncontrolled IOP serve
Patients group	C	4	63.0 ± 8.8	Underwent cataract extraction serve
Control group	—	4	50.5 ± 6.7	—

IOP, intraocular pressure.

## Data Availability

The data used to support the findings of this study are available from the corresponding author upon request.
